The article "Effect of exchange rate uncertainty, energy prices and sectoral spending on agriculture value added, household consumption, and domestic investment" was published in 2024. Journal: Heliyon.

# Effect of exchange rate uncertainty, energy prices and sectoral spending on agriculture value added, household consumption, and domestic investment

**DOI:** 10.1016/j.heliyon.2024.e30138

**Published:** 2024-04-23

**Authors:** Paul Terhemba Iorember, Nora Yusma Mohamed Yusoff, Philip Terhemen Abachi, Ojonugwa Usman, Andrew Adewale Alola

**Affiliations:** a Department of Economics, Nile University of Nigeria, Abuja, Nigeria; b UNITEN BUsiness School, Universiti Tenaga Nasional, Kajang 43000, Malaysia; c Department of Economics, Benue State University, Makurdi, Nigeria; d Department of Economics, Istanbul Ticaret University, Istanbul, Turkey; e Adnan Kassar School of Business, Lebanese American University, Beirut, Lebanon; f CREDS-Centre for Research on Digitalization and Sustainability, Inland Norway University of Applied Sciences, Norway; g Faculty of Economics, Administrative and Social Sciences, Nisantasi University, Istanbul, Turkey

**Keywords:** Exchange rate, Energy prices, Agriculture expenditure, Households consumption, Machine learning, Kernel regularized least squares

## Abstract

The agricultural value chain is underpinned by the interdependence of agricultural value added, household consumption and domestic investment. Understanding the complex interactions between these microeconomic outcomes and the uncertainties in the macroeconomic variables of exchange rates, energy prices and sectoral spending remains under-researched. Therefore, this study examines the impact of exchange rate, energy prices and sectoral spending on agricultural value added, household consumption and domestic investment in Nigeria from 1981 to 2020. Using Kernel regularized least squares (KRLS), the results show that the average pointwise marginal effects of exchange rate and agricultural spending are positive, while the average pointwise marginal effect of energy price is significantly negative for the agricultural value-added model. The results also show that the exchange rate, energy prices and agricultural expenditure all have a positive effect on household consumption. Regarding domestic investment, the effect of the exchange rate is positive and statistically insignificant, while the effects of energy prices and agricultural expenditure are negative and statistically significant. The study recommends the need to strengthen the social safety nets currently in place in Nigeria to support households that are vulnerable to exchange rate fluctuations. In addition, incentives should be given to households and farmers to help use renewable energy sources such as solar or wind power for agricultural activities. Also, investment in value chains and agribusiness initiatives should be encouraged rather than just in crop production.

## 1 Introduction

Globally, agriculture is regarded as a major determinant of economic prosperity in both developed and developing countries. It serves as a catalyst for economic and structural transformation, and provides the basis for economic diversification and sustainable development [1,2]. Agriculture also enables the proper utililization of countries' factor endowments, reduces the import demand for agriculturally based products, generates employment for the teeming population and increases foreign earnings through exports of agriculturally based products [2]. In Nigeria, the agricultural sector is the largest employer of labour, employing about 70 % of the workforce. This is despite several years of neglect and under-funding following the discovery of crude oil [3]. The agricultural value chain is underpinned by the interdependence of agricultural value added, household consumption and domestic investment. According to Zhang and Diao [4], these three elements are crucial in determining how the agricultural value chain behaves. The agricultural sector's contribution to the economy is reflected in agriculture value added. The entire amount of money spent by households on goods and services is referred to as household consumption. Household disposable income is influenced by the revenue from agricultural activities, including wages and profits [4]. Domestic investment includes money spent on infrastructure and capital goods inside a nation. According to Mouges et al. [5], domestic investment in agriculture can include money for irrigation systems, farm equipment, research and development (R&D), and other capital-intensive projects.

Currency exchange rates, energy prices and spending patterns of different sectors of an economy can have an impact on the interdependence of value-added agriculture, household consumption, and domestic investment. According to Sansika et al. [6], a decline in the value of the national currency can make agricultural exports more competitive in global markets. This may result in a rise in the market for agricultural goods, which would raise the value added to agriculture. Furthermore, if the value of the home currency declines, the cost of imported food may increase, which could lower household purchasing power and change consumption habits [6]. In the same way, changes in exchange rates may affect how much it costs to import capital goods and technologies for the agricultural industry [7]. Such imports could become more expensive due to a weakened currency, which could have an impact on decisions made about domestic investment.

Furthermore, energy is a major input in agriculture. It is used to power equipment, fertilizers, and serves as fuel. Farmers' cost of output goes up when energy prices rise. This may result in increased costs for running irrigation systems, farming equipment, and freight transportation. Increased energy costs could have an impact on how agricultural products are transported from farms to markets [8]. Elevated fuel prices may lead to increased shipping costs, which may affect the agriculture sector's total value added [9,10]. Similarly, household expenses for heating, power, and transportation are frequently raised by rising energy prices. As a result, there may be less money available for other products and services. Increasing energy costs may be a factor in the economy's overall inflation. Households may see a decline in purchasing power when the cost of essentials like food and transportation rises because of rising energy prices [11,12]. Also, certain sectors such as manufacturing and transportation may experience higher production costs because of rising energy prices. This may result in lower profit margins, which would restrict the amount of money available for domestic investment [13,14]. Higher energy costs, however, might encourage investment in renewable and alternative energy sources. Diversifying energy portfolios can encourage governments and corporations to invest more in greener and more sustainable energy solutions.

On the sectoral expenditure side, increased sectoral spending on agricultural infrastructure, such as storage facilities and irrigation systems, can boost agriculture value added by lowering post-harvest losses and increasing efficiency [2]. Similarly, higher investment in the agricultural industry can result in the creation of jobs and revenue [3]. This may have a favorable impact on household consumption levels and, in turn, spending patterns. Moreover, higher farm spending can boost agribusinesses and farm mechanization which focuses on raising the income of small-holder farm household through reduced production costs [15].

In Nigeria, successive governments since political independence in 1960 have focused on agriculture to diversify the economy, by designing and implementing several policies and programs. More recently, the Economic Recovery and Growth Plan (ERGP) prioritizes food security and aims to achieve self-sufficiency in tomato paste, rice, and wheat, by 2025 [16]. Furthermore, following the decline in revenue and reserves traceable to the oil crises of 2014 and 2015, the Central Bank of Nigeria (CBN) devalued the naira twice between November 2014 and February 2015 to mitigate the pressure on domestic currency, evident by the wide gap between the official and the parallel exchange rates [17]. These two episodes of devaluation, however, did not achieve the desired outcome. Next were the partial floating of the naira in June 2016 and the frequent intervention of the monetary authority (pumping of dollar in the exchange market). Similarly, to reduce imports and conserve its diminishing foreign exchange reserves, the CBN implemented a ban on access to foreign exchange at the CBN official window for a list of 41 items. This list includes rice, poultry, and palm oil products [17]. Additionally, the Federal Government increased import levies on these goods and other agricultural products, and even banned imports of some of these items entirely [17]. More recently, the Central Bank of Nigeria has removed the rate cap on the domestic currency (naira) at the official window of the foreign exchange market, allowing for a free float of the national currency against the dollar and other global currencies.

Nigeria's government has also prioritized spending on agriculture because of the sector's significance to the nation's economy. In addition to promoting economic growth and food security, agriculture is a major employer. Generally, the Nigerian government provides funding for a range of agricultural projects, programs, and subsidies to assist farmers, boost output, and deal with issues facing the industry. Despite these policy interventions, the agriculture sector remains underdeveloped, primarily because the focus has been on production, rather than on enhancing domestic value-addition across the value chain segments. For instance, an analysis from cocoa barometer suggests that in the production of a bar of chocolate, a marginal 6.6 % of the value-added is in the production, while the remaining is in the processing, marketing, and retail segments of the value chain which directly involve household consumption and domestic investment [18]. Based on the context outlined above, this study explores the effect of exchange rate uncertainty, energy prices and sectoral spending on agriculture value added, household consumption, and domestic investment in Nigeria.

Our research makes the following contributions to the existing literature. First, this study deepens the knowledge of the complex interactions between macroeconomic variables (exchange rates and sectoral spending) and microeconomic outcomes (agriculture value added, household consumption and domestic investment). It clarifies how adjustments made at the macro level affect the economy down to the micro level. Second, the research fosters a cross-disciplinary knowledge of the intricate dynamics at play by incorporating insights from agricultural studies, finance, and economics. This multidisciplinary method helps to provide a more thorough and sophisticated understanding of the economic system. Third, the study applies the KRLS machine learning algorithm which permits the handling of regression and classification issues without making robust functional form assumptions or doing a manual specification search. By leveraging KRLS, the study uses data-driven analytics to find hidden patterns and linkages in the data. As a result, decision-makers and other interested parties might be better equipped to base their plans and actions on empirical knowledge.

The rest of the paper is sectionalized as follows: Section 2 focuses on a brief literature review involving theory and empirical reviews. Section 3 deals with materials and methods. Section 4 presents results and discussion, and Section 5 concludes the study.

## 2 Literature review

Theoretically, the effectiveness of devaluation depends on the Marshall-Lerner condition, which states that when the sum of price elasticity of the demand for imports of any two countries trading their goods between themselves is greater than unity, devaluation tends to increase exports, and decrease imports [19]. This may not be said of the Nigerian economy that is largely import-dependent and mono-product for many years. Also, according to the speculations of the J-curve relationship, every economy passes through periods of weak growth in the early phase of devaluation policy but with sound implementation strategies, mixed with sound fiscal policies such as increased agriculture spending, the economy returns to the path of increasing growth in the long run [20]. However, the period it takes to achieve sustainable growth varies among different countries.

Furthermore, the literature regarding the impact of exchange rate variations on output is enormous but very little has been done concerning the impact of the policy changes on agricultural investment demand, households’ consumption, and income. For example, Orji et al. [21] examine the impact of exchange rates on sectoral value addition and sustainable economic growth in the Economic Community of West African States (ECOWAS) via the monetary policy channel from 2013 to 2019. Applying the fixed-effect OLS with Driscoll–Kraay, the results showed that the impact of exchange rate on the value added of the agricultural sector is primarily heterogeneous and significantly in-elastic. Nwalem et al. [22] investigates effect of investment and exchange rate on agricultural output (groundnut production) in Nigeria using data from 1980 to 2016. Applying the vector error correction model, the study showed that both exchange rate and public agriculture spending contribute 0.3 % each to groundnut output in Nigeria. Similarly, Asaleye et al. [1], in a study on the effect of selected macroeconomic variables on agricultural output in Nigeria, found a positive and statistically significant relationship between exchange rate and agricultural sector output. Eche et al. [23] investigate how household consumption expenditures in African emerging economies are adjusted to variations in exchange rates. The study uses the modified versions of non-linear autoregressive distributed lag (ARDL) and multiple threshold non-linear ARDL, which specifically illustrates how distinct, positive, and negative fluctuations in explanatory variable(s) impact on the dependent variable.

Thus, the empirical estimates show that, except for Nigeria, the impacts of exchange rate fluctuations on consumption spending vary across country. Njindan et al. [24] investigate how Ghanaian consumption is impacted by fluctuations in exchange rates. The annualized variance of the real exchange rate, which serves as a gauge of exchange rate volatility, was calculated using yearly data from 1980 to 2015. The results demonstrate that exchange rate volatility has short-term negative effects on domestic consumption that carry over into long-term negative effects. Earlier research by Bahmani-Oskooee et al. [25] also supports the idea that while exchange rate uncertainty affects domestic consumption in practically every country in the short term, only half of those effects persist over the long term. Siddig [26] uses an economy-wide impact assessment tool to investigate the possible effects of devaluing the overvalued. Similarly, Eltalla [27] analyses the impacts of the devaluation on the Palestinian economy using computable general equilibrium model on the 2012 social accounting matrix for Palestine. The study finds that a 15 % devaluation of the exchange rate reduces real gross domestic product by 1.99 %, while it declines import and export by 20.61 % and 52.67 % respectively. Also, 15 % devaluation reduces the level of private consumption by 6.31 % and increases inflation by 4.7 %.

Regarding the effect of energy prices, Ma et al. [9] examine the role of energy prices in influencing agricultural production, and energy consumption in China using the price endogenous partial equilibrium model analysis. The results show that higher energy prices reduce producers’ welfare and diminish agricultural energy consumption. In a study on the price and income elasticities of residential energy demand in Germany, Schulte and Heindl [11] find that fluctuations in energy prices affect households with lower incomes more than those with higher incomes. By distinguishing between the demand for heating and electricity, Reaños and Wölfing [12] investigate the distributional consequences of growing energy prices for households. The findings show that price rises for heating are more regressive than those for electricity. Mallick et al. [13] endogenize public sector investment to investigate the effect of the international crude oil price on private investment in India using annual data covering the years 1980–2014. Based on empirical estimation, the study shows that the growth of domestic private investment in India is negatively impacted by both the price of crude oil and the level of investment.

Regarding agricultural sector spending and output growth [3,19,28,29], establish that agriculture expenditure has a positive relationship with output growth while the study of [30] reveals a negative relationship between agricultural spending and output growth. Concerning household income/welfare [1,2], establish that increasing government agricultural spending would bring about an increase in households’ income and subsequently improve general well-being. Furthermore, studies by Refs. [31,32] find that exchange rate have negative effect on agricultural output in Nigeria. While the study by Ref. [33] find that currency devaluation has led to significant increases in costs of major agricultural inputs over the last two years, which influence costs of agricultural outputs across the value chain in the Niger Delta region of Nigeria.

The interaction of energy costs, sectoral spending, exchange rate uncertainty, and their impact on domestic investment, household consumption, and agriculture value added is a complex area of economic study. A survey of the empirical literature revealed a dearth of studies examining the interactions between these variables in particular geographic contexts, particularly in developing nations or understudied areas like Nigeria. Due to variations in economic structures, reliance on energy, and agricultural methods, the effects of exchange rate volatility and energy prices can range greatly between nations. Not enough is known about the dynamic and potentially nonlinear relationships that occur over time between sectoral spending, energy prices, and exchange rate uncertainty. To create successful policy interventions and predicting future trends, it is essential to comprehend these processes.

## 3 Data and methods

### 3.1 Data

This study utilizes annual time series data over the period 1981–2020, based on data availability. Table 1 presents the variables, definition, measurement, and sources of data used in the study.

**Table 1:** Definition, measurement and sources of variables.

Variables	Definition and measurement	Sources
AgVA	Agriculture Value Added (Agriculture, forestry, and fishing, value added as percentage of GDP)	World Development Indicators (WDI) - https://databank.worldbank.org/source/world-development-indicators
HHC	Household Consumption (Households and NPISHs^a^ final consumption expenditure as percentage of GDP)	WDI -https://databank.worldbank.org/source/world-development-indicators
DINV	Domestic Investment (Gross fixed capital formation as percentage of GDP)	WDI - https://databank.worldbank.org/source/world-development-indicators
EXR	Exchange Rate (Official LCU–naira per US Dollar)	WDI - https://databank.worldbank.org/source/world-development-indicators
EP	Energy Price Inflation	World Bank - https://www.worldbank.org/en/research/brief/inflation-database
GEA	Government Expenditure on Agriculture	Central Bank of Nigeria (CBN) - https://www.cbn.gov.ng/documents/Statbulletin.asp
GEE	Total Government Expenditure on Education	CBN - https://www.cbn.gov.ng/documents/Statbulletin.asp

a Non-profit institutions serving households.

### 3.2 Modeling procedure and estimation techniques

In this paper, we construct the following stochastic econometric models to investigate the effects exchange rate and agricultural sector spending on agricultural value added, household consumption and domestic investment.

(1) $$AgVA_{t}=\alpha_{0}{\left(AgVA\right)}_{t-i}+\alpha_{1}{\left(EXR\right)}_{t}+\alpha_{2}{\left(EXR\right)}_{t-i}+\alpha_{3}{\left(EP\right)}_{t}+\alpha_{4}{\left(EP\right)}_{t-i}+\alpha_{5}{\left(GEA\right)}_{t}+\alpha_{6}{\left(GEA\right)}_{t-i}\alpha_{7}{\left(GEE\right)}_{t}+\alpha_{8}{\left(GEE\right)}_{t-i}+\varepsilon_{t}$$

(2) $$HHC_{t}=\beta_{0}{\left(HHC\right)}_{t-i}+\beta_{1}{\left(EXR\right)}_{t}+\beta_{2}{\left(EXR\right)}_{t-i}+\beta_{3}{\left(EP\right)}_{t}+\beta_{4}{\left(EP\right)}_{t-i}+\beta_{5}{\left(GEA\right)}_{t}+\beta_{6}{\left(GEA\right)}_{t-i}\beta_{7}{\left(GEE\right)}_{t}+\beta_{8}{\left(GEE\right)}_{t-i}+\varepsilon_{t}$$

(3) $$DINV_{t}=\varphi_{0}{\left(DINV\right)}_{t-i}+\varphi_{1}{\left(EXR\right)}_{t}+\varphi_{2}{\left(EXR\right)}_{t-i}+\varphi_{3}{\left(EP\right)}_{t}+\varphi_{4}{\left(EP\right)}_{t-i}+\varphi_{5}{\left(GEA\right)}_{t}+\varphi_{6}{\left(GEA\right)}_{t-i}\varphi_{7}{\left(GEE\right)}_{t}+\varphi_{8}{\left(GEE\right)}_{t-i}+\varepsilon_{t}$$

Where $\alpha_{0}$, $\beta_{0}$, $\varphi_{0}$ are the coefficients of the lag dependent variables as shown in equations (1), (2), (3) respectively. $\alpha_{1}$- $\alpha_{8}$, $\beta_{1}$- $\beta_{6}$, and $\varphi_{1}$ - $\varphi_{8}$ are the parameter estimates of the respective models. The variables remain as earlier defined in Table 1. In addition to the main explanatory factors, we add education spending as a control variable. Since education can have significant and far-reaching effects on household consumption, domestic investment, and agricultural value added, it is imperative to account for education spending in models relating to these economic variables. People's human capital is improved via education. Since educated people are more likely to use contemporary, effective farming methods as well as different patterns of consumption and investment, controlling for education expenditure helps separate the effects of human capital on agricultural value added, household income, and domestic investment [34].

To estimate the model coefficients in Equations (1), (2), (3)), we use the Kernelized Regularized Least Squares (KRLS) method which was developed by Hainmueller and Hazlett [35] and Ferwerda et al. [36] for social science-based modeling and inference problems. The KRLS is a machine learning algorithm that combines the principles of regularized least squares regression with kernel methods. It is often used for regression tasks, where the objective is to predict a continuous output variable based on input information [35].

The KRLS utilized in this study employs a potent regression technique that blends regularized least squares regression with kernel methods concepts. The selection of the KRLS model is motivated by multiple benefits. Firstly, it allows users to deal with problems related to regression and classification without having to perform a manual specification search or make strong assumptions about the functional form. Unlike the other methodologies, the KRLS methodology addresses regression and classification problems without necessarily considering the additivity and linearity assumptions [37]. Additionally, the method's avoidance of strong parametric assumptions makes it appropriate for social science investigations. Based on the idea that factor variables with nearly similar values should, on average, produce results that are comparable, the KRLS estimator covers a much wider range of possible functions. The KRLS's regularization concept also enables it to quantify fragility and volatility, reduce overfitting, and lessen the effects of poor leverage points.

Moreover, the KRLS estimator has favorable statistical properties including unbiasedness and consistency. It is robust to classification and multicollinearity problems such as functional form and misspecification bias often associated with least squares and generalized linear models. Since the KRLS offers the marginal effects of each component variable on the dependent variable across units, it takes non-linearity issues into account (i.e., at each data point). The KRLS is suitable for modeling problems like model-based causal inference, prediction problems, exploratory analysis, and other regression and/or classification problems when the precise functional form is unknown [35,36,38]. We can evaluate the marginal impacts of each component variable on the dependent variable across units using the KRLS approach, in general.

For robustness, we apply the novel dynamic ARDL (DYNARDL) simulation approach by Refs. [39,40]. The DYNARDL simulation approach is applied in a straightforward but technical manner. First, a stringent first-difference stable I(1) dependent variable is necessary for the DYNARDL simulation approach [40,41]. Second, the variables must be cointegrated and a dependent variable that is non-stationary at level I(0) is a potential requirement for cointegration. To determine the cointegration or long-term link among the variables, we apply the limits test within the framework of the Autoregressive Distributed Lag (ARDL) model [42]. Both the F-statistics and the t-statistic must be higher than their corresponding hypothesized values at a particular level of significance (5 % in this study) for the ARDL bounds testing technique to cointegration to be valid. Compared to other traditional cointegration tests, the bound testing method has some benefits. The small sample advantage is one of the advantages; it produces consistent findings even with a tiny sample size. Also, the method can be used whether the series are all I(0)s, I(1)s, or are fractionally integrated [39,[43], [44], [45]]. The generic ARDL (p, q, …, q) is updated in accordance with Kripfganz and Schneider [46] to take into consideration the influence of additional elements as:

(4) $$Y_{t}=\alpha_{0}+\sum_{i=1}^{k}\beta_{i}Y_{t-i}+\sum_{i=0}^{l}\gamma_{i}^{\prime }X_{t-i}+\sum_{i=0}^{l}\varphi_{i}^{\prime }Z_{t-1}+\mu_{t}$$

Where $Y_{t}$ in equation (4) stand for the dependent variable(s), $X_{t}$ is a column vector of the main independent variables (exchange rate and agriculture expenditure); $Z_{t}$ is a vector of the control variable (education expenditure); β, γ and φ are the coefficient estimates, α is the intercept term and μ is the independent and identically distributed (i.i.d) white noised error term.

For the unit root properties of the variables, we use the standard Augmented Dickey Fuller (ADF) test without breaks and the modified ADF test with one break point to assess this conditional requirement. According to Nwani et al. [47], the two variations of the break point test, Innovative outlier (IO) and additive outlier (AO) are used. Whereas the AO modified ADF break point test views structural break as an instantaneous event, the IO version of the modified ADF break point test views structural break as a progressive occurrence. The three ADF tests compare the alternative hypothesis that the series is stationary to the null hypothesis that it follows a unit root process and is non-stationary [47].

Fig. 1 shows the stages of the empirical analysis employed in this study.

**Fig. 1:** Flow chart analysis.

## 4 Results and discussion

### 4.1 Descriptive statistics

Table 2 provides the descriptive statistics of the variables and correlation analysis between variables. Starting from the descriptive statistics, we find that mean of the variable are close to each other with HHC having the largest mean score of 3.9195 while GEA has the smallest mean score of 1.004. Furthermore, the standard deviation of AGVA, HHC, DINV, and EP is less than 1, suggesting that these variables are less volatile. However, for EXR, GEA, and GEE, we find that the standard deviation is 1.9930, 2.9601, and 2.8205. The implication of high standard deviation is that the distribution of these variables has more variability, which is perhaps different from the means, i.e. the data is not clustered around the mean of the distribution. Also, apart from DINV and EP, all the variables are skewed negatively with HHC exhibiting large skewness value. The kurtosis is positive for all variables with AGVA, HHC, and EP displaying a large value, which signifies a leptokurtic distribution while the rest of the variables exhibit a platykurtic distribution. However, the null hypothesis for normal distribution is rejected only for the case of HHC at 5 % level of significance.

**Table 2:** Descriptive statistics.

	AGVA	HHC	DINV	EXR	EP	GEA	GEE
Mean	3.1091	3.9195	3.4423	3.5403	2.7612	1.0045	2.9571
Median	3.0942	4.0540	3.4651	4.6720	2.7131	1.9875	3.9175
Maximum	3.6100	4.4010	4.4930	5.8828	5.3771	4.2524	6.3859
Minimum	2.5047	2.2859	2.6510	−0.4943	0.7419	−4.3607	−1.8192
Std. Dev.	0.2098	0.4567	0.5261	1.9930	0.8781	2.9601	2.8205
Skewness	−0.5644	−2.0028	0.0721	−0.7973	0.6056	−0.6457	−0.5153
Kurtosis	4.5108	7.2465	2.0750	2.3583	4.0097	1.9841	1.8429
Jarque-Bera	5.9280	56.7971	1.4608	4.9242	4.1438	4.4992	4.0016
Probability	0.0516	0.0000	0.4817	0.0853	0.1259	0.1054	0.1352

### 4.2 Unit root tests without and with structural breaks

To ensure the validity of the results and prevent erroneous conclusions, it is essential to evaluate the stationarity status of the variables being examined. To achieve this, we use the augmented Dickey-Fuller test without structural break and with modification and structural break and the results are in Table 2. Panel X of Table 3 shows the results of the conventional ADF test, while Panels Y and Z show the results of the Innovative Outliers (IO) and Addictive Outliers (AO) variants of the modified ADF breakpoint test. The result in panel X makes it abundantly clear that each research variable has a unit root at level. However, according to their first difference, the nonstationary variables become stationary, indicating that the series in the model are I(1) processes. In the presence of structural breaks, the ADF test loses strength and yields inaccurate results. To achieve a single structural break point, the ADF test is modified utilizing IO and AO. After taking into account the structural break in the series, the findings in panels Y and Z confirm that all the variables are I(1). It is evident that throughout the chosen break years, the country experienced some significant policy shocks and upheavals. Overall, the results of the modified ADF unit root test with structural break support the use of ARDL, as they show that the data series are I(1), with no evidence of I(2) processes.

**Table 3:** Unit root tests using ADF and Modified ADF with One Structural Break Point.

	at Level form I(0)		at First Difference I(1)		
	t-Statistic	Break Date	t-Statistic	Break Date	Integration
Panel X: Augmented Dickey-Fuller (ADF) test					
AgVA	−2.138	–	−6.293***	–	I(1)
HHC	−2.122	–	−5.419***	–	I(1)
DINV	−2.186	–	−4.611***	–	I(1)
EXR	−2.109	–	−5.293***	–	I(1)
EP	−4.007	–	−7.836***	–	I(1)
GEA	−2.124	–	−8.688***	–	I(1)
GEE	−2.275	–	−7.886***	–	I(1)
**Panel Y: Modified ADF with one structural break point - Innovative Outlier (IO) test**					
AgVA	−3.949	2002	−7.628***	2002	I(1) with a break
HHC	−3.313	2000	−8.905***	1985	I(1) with a break
DINV	−2.946	1999	−6.300***	2017	I(1) with a break
EXR	−3.556	1985	−7.874***	1999	I(1) with a break
EP	−4.524	2006	−8669***	1991	I(1) with a break
GEA	−2.457	1986	−10.740***	1999	I(1) with a break
GEE	−3.107	1992	−9.022***	1992	I(1) with a break
**Panel Z: Modified ADF with one structural break point - Additive Outlier (AO) test**					
AgVA	−4.108	2002	−7.379***	2005	I(1) with a break
HHC	−3.797	2000	−9.146***	1985	I(1) with a break
DINV	−2.776	1999	−6.747***	2017	I(1) with a break
EXR	−3.184	1985	−6.109***	2001	I(1) with a break
EP	−4.983	1994	−8.669***	1991	I(1) with a break
GEA	−2.464	1986	−9.305***	2008	I(1) with a break
GEE	−2.618	1999	−8.298***	1988	I(1) with a break

Note: ***, ** and * indicate rejection of the null hypothesis at 1 %, 5 % and 10 % levels respectively.

### 4.3 Effects of exchange rate and agriculture sector expenditure on agriculture value added, household consumption and domestic investment

To evaluate the effects of exchange rate, energy prices and agriculture sector expenditure on agriculture value added, household consumption and domestic investment, we apply the KRLS procedure and the results are shown in Table 4 and Fig. 2, Fig. 3, Fig. 4. Table 4 displays the pointwise derivatives of the estimated KRLS for the three models. For model 1, the results show a prediction power of 0.7365 implying that the independent variables account for 73.65 % of the variations in agriculture value added. The 25th, 50th, and 75th percentiles show the analysis of the heterogeneous marginal effects using the independent variables derivatives. The robustness of the pointwise derivatives is confirmed by the absence of any evidence of diverse marginal effects across the chosen variables. Further, the average pointwise marginal effects of exchange rate, energy prices, agriculture expenditure and education expenditure are observed to be 0.0769 %, −0.0285 %, 0.0044 % and −0.0179 %, respectively. This shows the influence of the independent variables on agricultural value added. Specifically, the results imply that devaluation of the national currency can make a country's agricultural products more competitive on world markets [21]. This is because a weaker currency reduces the cost of domestic goods in terms of foreign money, which could increase agricultural exports. As farmers benefit from larger markets, this can ultimately lead to an increase in the value added by agriculture. Increased export earnings can have a positive impact on agricultural value added. Foreign consumers may find the country's agricultural products more affordable as the local currency weakens, thereby increasing demand and raising the income of agricultural producers.

**Table 4:** Pointwise derivatives using KRLS.

Parm	Avg	SE	t	p > |t |	P25	P50	P75
**Model 1**							
EXR	0.0769	0.0159	4.835	0.001	−0.1232	−0.0507	0.6480
EP	−0.0285	0.0103	−2.775	0.032	−0.0272	−0.0148	0.0221
GEA	0.0044	0.0250	0.175	0.862	−0.0173	0.0088	0.0258
GEE	−0.0179	0.0109	−1.646	0.108	−0.0585	−0.0294	0.0258
**Diagnostic**							
*Lambda*	*0.2935*	*Sigma*	*4*	*R*^*2*^	*0.7365*		
*Tolerance*	*0.04*	*Eff.df*	*10.07*	*Looloss*	*3.479*		
**Model 2**							
EXR	0.1107	0.0542	2.041	0.049	0.0505	0.0815	0.1035
EP	0.3227	0.0647	4.989	0.000	−0.1311	0.0686	0.6833
GEA	0.0340	0.0347	0.981	0.333	−0.0041	0.0183	0.0720
GEE	0.0493	0.0360	1.370	0.179	0.0374	0.0525	0.0652
**Diagnostic**							
*Lambda*	*0.010758*	*Sigma*	*4*	*R*^*2*^	*0.7772*		
*Tolerance*	*0.04*	*Eff.df*	*13.22*	*Looloss*	*8.117*		
**Model 3**							
EXR	0.0467	0.0427	1.094	0.281	0.0125	0.1326	0.1326
EP	−0.2718	0.0454	−5.987	0.000	−0.1187	0.0589	0.6519
GEA	−0.0069	0.0276	−0.253	0.802	−0.0057	0.0238	0.0238
GEE	0.1530	0.0285	−5.363	0.000	−0.1215	−0.0705	−0.7005
**Diagnostic**							
*Lambda*	*0.5518*	*Sigma*	*4*	*R*^*2*^	*0.9402*		
*Tolerance*	*0.04*	*Eff. df*	*15.33*	*Looloss*	*3.212*		

Note: Model 1 - agricultural value added, Model 2 – household consumption and Model 3 – domestic investment. Avg – average pointwise marginal effect, SE – standard error.

**Fig. 2:** **(a, b, c, d):** Pointwise marginal effect of exchange rate, energy prices, agriculture expenditure and education expenditure against agriculture value added.

**Fig. 3:** **(e, f, g, h):** Pointwise marginal effect of exchange rate, energy prices, agriculture expenditure and education expenditure against household consumption.

**Fig. 4:** **(I, j, k, i):** Pointwise marginal effect of exchange rate, energy prices, agriculture expenditure and education expenditure against domestic investment.

Contrary to popular belief, a country's greatest interests are not always served by a strong currency. A country's exports become more competitive on international markets, while imports become more expensive when the domestic currency is weak. Increased export volumes and expensive imports both contribute to economic growth because customers choose domestic alternatives to imported goods [48]. This translates into improvements in terms of trade, quicker economic growth, and increased employment. Our finding is consistent with those of [49,50], who establish that a change in exchange rate is associated with an increase in output growth in Nigeria and South Africa. Also, our finding concurs with [51], who finds that changes in exchange rates cause upward variations in the growth of BRICS economies.

Further, increasing energy prices raise the cost of transportation. Since transportation of goods from farms to markets, distribution hubs, and processing facilities is a part of agriculture, an increase in fuel prices might result in higher transportation costs. This may result in higher costs for farmers to promote their goods, which would lower their total profitability and weaken overall productivity. Similarly, the cost of agricultural inputs rises along with energy prices. Fuel, electricity, and other energy-dependent input costs may increase for farmers, which could lower their profit margins. This finding aligns with the findings of [9,10] Also, increasing funding for agricultural R&D can result in the creation of new technology, enhanced crop types, and more productive farming methods. These developments have the potential to boost yields, improve productivity, and advance the agricultural industry. Additionally, the efficiency of the agricultural supply chain can be raised by making investments in infrastructure related to agriculture, such as storage facilities, rural roads, and irrigation systems. This may lead to decrease in post-harvest losses, reduction in transportation expenses, and ensures efficiency in getting agricultural products to market.

For models 2 and 3, the results showed the prediction powers of 77.72 % and 94.04 % respectively. The robustness of the pointwise derivatives is confirmed by the absence of the diverse marginal effects across the chosen variables in both models as shown in 25th, 50th, and 75th percentiles. Similarly, the demonstrable influence of exchange rate, energy prices, agriculture expenditure and education expenditure are observed to be 0.1107 %, 0.3227 %, 0.0340 % and 0.0497 %, respectively for model 2, and 0.0467 %, 0.2718 %, 0.0069 % and 0.1530 % respectively for model 3.

Regarding the household consumption effect in model 2, the results suggest that if the value of the home currency drops, the cost of imported goods may increase, driving up family expenses. Moreover, a weaker currency can make inflationary pressures worse by driving up the cost of imported goods and services, which could in turn reduce real income and reduce the purchasing power of household income. More so, the cost of producing agricultural products can go up with rising energy prices, especially when it comes to energy-intensive tasks like transportation, irrigation, and machine operation. Farmers' profitability and, consequently, household income and consumption may suffer as a result. Increased energy costs may have an impact on allied industries like agro-processing and transportation in addition to farming operations in rural areas where agriculture is a major source of income. This may have an impact on rural income. Furthermore, if more money is spent on infrastructure, support services, research and development, and other aspects of agriculture, it can boost output. Increased yields, greater revenue for farmers, and a favorable effect on household income can all result from enhanced productivity. This finding is consistent with the findings of [[11], [12], [13]] which showed that higher energy prices are regressive with respect to household income.

Moreover, the results suggest that increasing government spending on an important sector such as agriculture will boost economic activity and improve household welfare. As spending on agriculture increases, more resources become available to add value to agricultural products. This finding agrees with [2,52,53] who also document that increasing expenditure in agriculture is positively associated with an increase in households’ income and the general well-being of households. The finding is however contrary to the finding of Takeshima & Liverpool-Tasie [15] which show that government spending on fertiliser subsidies in Nigeria has had relatively limited effects on agricultural and food commodity prices. This is partly because the domestic food market and food imports are relatively well integrated, and sometimes tariffs on imported food have the effect of raising local food prices. A higher price would be costly to consumers and could have a negative impact on consumption, although it could benefit some producers.

Concerning domestic investment effect in model 3, the results reveal that a country's exports become more competitive when its own currency depreciates, which could stimulate industries that are focused on exports. Thus, economic activity and domestic investment may be boosted, especially in industries with an eye toward global markets. Conversely, a depreciating currency may make imported capital goods and raw commodities more expensive. This may make production more expensive for home companies, which would discourage investment in some sectors of the economy. Furthermore, changes in energy prices can have an immediate effect on a company's cost of production, particularly if that company operates in an energy-intensive industry. Elevated energy costs can escalate operational costs, hence diminishing profit margins and, occasionally, discouraging investment. Similarly, large government spending on agriculture can increase competition for available funds, especially if it is supported by borrowing. This could lead to higher interest rates and discourage private investment in other areas by making it more expensive for businesses to borrow money. If too many resources are devoted to agriculture, money may be taken away from more lucrative and dynamic industries such as manufacturing, services, or technology. The overall diversity and growth of the economy can be hampered by this misallocation.

Further, we look at how changes in exchange rate, energy prices and agriculture expenditure over time impact agriculture value added, household consumption and domestic investment. To capture the various marginal effects, we plot the pointwise derivatives of exchange rate, energy prices and agriculture expenditure against agriculture value added, household consumption and domestic investment, and the results shown in Fig. 2, Fig. 3, Fig. 4 respectively. Evidently, Fig. 2 (a, b, c, d) show that higher levels of exchange rate, energy prices and agriculture expenditure increase agriculture value added at the lower levels. However, the rate of change decrease with time across all the factors except for education which serves as a control variable in the study. This suggests that exchange rate, energy prices and agriculture expenditure have increasing marginal returns on agriculture only to a certain level. This explains the plausibility of ensuring a stable exchange rate and constantly reviewing agriculture expenditure to avoid rebound effect afterward. Fig. 3 (e, f, g, h) depicts that the marginal effect of exchange rate and agriculture expenditure on household consumption became higher with time, while the marginal effects of energy prices and education expenditure decline with the passage of time. In Fig. 4 (i, j, k, l) the results indicate that the marginal effects of all the factors (exchange rate, energy prices and agriculture expenditure) on domestic investment decrease over time. In effect, fluctuations in energy costs, exchange rates, and agricultural spending can all lead to difficult economic conditions that have an impact on the confidence and profitability of enterprises. All of these reasons together may cause businesses to become less willing to invest in new ventures or expansions, which in turn may lead to a decline in domestic investment.

### 4.4 Robustness

To verify the robustness of the KRLS machine learning results in Table 4 and Fig. 2, Fig. 3, Fig. 4, we apply the DYNARDL simulation model, and the results are summarized in Table 5 (panels A and B) and Fig. 5, Fig. 6, Fig. 7. First, Table 5 Panel A presents the results of the ARDL bounds tests. The results also include a summary of the vector autoregressive (VAR) lag order selection criteria. Table 5 Panel B shows the Kripfganz and Schneider [46] critical values and approximate p-values. The estimated F- and t-statistics in panel A are compared with the critical values from Kripfganz and Schneider [46] in Panel B to decide on the existence of cointegration in the models. This approach is robust to the small sample size structure of the time series. The results show evidence of cointegration between the variables in all the three estimated models. For each model, the F- and t-statistics are above the upper critical limit at the 5 % significance level. This means that the null hypothesis of no cointegration is rejected for all the three models. The results of the bounds test thus support the existence of a long-run relationship between the variables over the course of the study.

**Table 5:** ARDL-Bounds cointegration with Kripfganz and Schneider [46] critical values.

		Model 1 AgVA	Model 2 HHC	Model 3 DINV
Panel A: ARDL Bounds				
Selected Model		ARDL(3, 0, 3, 4)	ARDL(1, 0, 3, 0)	ARDL(1, 0, 3, 0)
Lag Selection		AIC	AIC	AIC
Break		2002	2000	1999
F-Statistic, F		5.532**	6.605**	4.947*
t-Statistic (t)		−4.964**	−4.614**	−3.882*
Panel B: Kripfganz and Schneider [46] critical values and approximate p-values				
1 % critical values				
I(0)	F (t)	5.228 (−3.639)	5.179 (−3.636)	5.154 (−3.634)
I(1)	F (t)	7.330 (−4.718)	6.937 (−4.673)	6.740 (−4.650)
5 % critical values				
I(0)	F (t)	3.546 (−2.860)	3.587 (−2.906)	3.608 (−2.929)
I(1)	F (t)	5.126 (−3.828)	4.961 (−3.851)	4.878 (−3.862)
10 % critical values				
I(0)	F (t)	2.844 (−2.483)	2.926 (−2.550)	2.956 (−2.584)
I(1)	F (t)	4.226 (−3.395)	4.131 (−3.446)	4.084 (−3.471)

Note: ***, ** and * denote rejection of H_0_ of no cointegration at 1 %, 5 % and 10 % respectively. Reject Ho if both F and t are more extreme than critical values for I(1) variables.

**Fig. 5:** **(m, n, o):** Plots of the dynamic simulated ARDL model representing counterfactual shock in predicted exchange rate (EXR). Black dots (●) are the predicted respective agriculture value added (AgVA), household consumption (HHC) and domestic investment (DINV) by 1 % shock in EXR; thick black, light black and light-blue spikes denote 75, 90, and 95 % confidence interval. (For interpretation of the references to colour in this figure legend, the reader is referred to the Web version of this article.)

**Fig. 6:** **(p, q, r):** Plots of the dynamic simulated ARDL model representing counterfactual shock in predicted energy prices (EP). Black dots (●) are the predicted respective agriculture value added (AgVA), household consumption (HHC) and domestic investment (DINV) by 1 % shock in EP; thick black, light black and light-blue spikes denote 75, 90, and 95 % confidence interval. (For interpretation of the references to colour in this figure legend, the reader is referred to the Web version of this article.)

**Fig. 7:** **(s, t, u):** Plots of the dynamic simulated ARDL model representing counterfactual shock in predicted government expenditure on agriculture (GEA). Black dots (●) are the predicted respective agriculture value added (AgVA), household consumption (HHC) and domestic investment (DINV) by 1 % shock in GEA; thick black, light black and light-blue spikes denote 75, 90, and 95 % confidence interval. (For interpretation of the references to colour in this figure legend, the reader is referred to the Web version of this article.)

Having confirmed cointegration in all the three models, the study applies the dynamic simulated ARDL to capture the long-term impact of counterfactual shocks in the factor variables on agriculture value added, household consumption, and domestic investment, and the results are presented in Fig. 5, Fig. 6, Fig. 7. Specifically, Fig. 5 (m, n, o) presents the responses of agriculture value added, household consumption, and domestic investment to a counterfactual shock in the predicted exchange rate (EXR). The results show that a 1 % shock in the predicted exchange rate affects agriculture value added and household consumption in the first period, but growth accelerates afterward, while the effect on domestic investment appears to be stable over time. Fig. 6 (p, q, r) captures the counterfactual shocks in the predicted energy prices. It reveals that a 1 % shock in predicted energy prices accelerates growth in agriculture value added and decreases growth in domestic investment after the first period. However, the effect on household consumption appears to be relatively stable. Fig. 7 (s, t, u) shows the counterfactual shock in predicted government expenditure on agriculture value added, household consumption, and domestic investment. Evidently, the results indicate that a 1 % shock in predicted agriculture expenditure has a negligible depressing impact on agriculture value added, household consumption, and domestic investment. This finding aligns with the reality in Nigeria, where agricultural spending may not always be distributed properly or efficiently. Funds may not be used to their full potential or may not reach the intended beneficiaries due to poor planning, corruption, or mismanagement. More so, Nigeria has infrastructural issues such as roads and irrigation systems that may reduce the return on agricultural spending [2,3]. The robustness test results, akin to the KRLS results, indicate that fluctuations in exchange rates, energy prices, and agriculture spending do not have a permanent effect on the target variables; hence, policy alternatives should be continuously reviewed.

## 5 Conclusion and recommendations

This study examines the effect of exchange rate uncertainty, energy prices and agriculture expenditure on agriculture value added, household consumption and domestic investment in Nigeria over the period 1981 to 2020. Applying Kernel-based Regularized Least Square, the results suggest that the average pointwise marginal effects of exchange rate and agricultural expenditure are positive, while the average pointwise marginal effect of energy price is negative. This shows the influence of the independent variables on agricultural value added. This means that the positive effect (depreciation) of the national currency can make a country's agricultural products more competitive on world markets. This is because a weaker currency reduces the cost of domestic goods in terms of foreign currency, which could increase agricultural exports. Similarly, increased funding for agricultural R&D can lead to the development of new technologies, improved crop varieties and more productive farming methods. These developments have the potential to increase yields, improve productivity and advance the entire agricultural industry. In addition, investments in agricultural infrastructure, such as storage facilities, rural roads, and irrigation systems, can improve the efficiency of the agricultural supply chain. However, rising energy prices are increasing transport costs. As part of agriculture is the transport of goods from farms to markets, distribution centres and processing plants, an increase in fuel prices can lead to higher transport costs. This may result in higher costs for farmers to transport their goods, which would reduce their profitability and weaken overall productivity.

For household consumption, the results show that if the value of the home currency drops, the cost of imported goods may increase, driving up family expenses. Moreover, a weaker currency can make inflationary pressures worse by driving up the cost of imported goods and services, which could in turn reduce real income and reduce the purchasing power of household income. Similarly, increased energy costs may have an impact on allied industries like agro-processing and transportation in addition to farming operations in rural areas where agriculture is a major source of income. This may have an impact on the entire rural income. Furthermore, if more money is spent on infrastructure, support services, research and development, and other aspects of agriculture, it can boost output. Increased yields, greater revenue for farmers, and a favorable effect on household income can all result from enhanced productivity.

Concerning domestic investment effect, the findings reveal that a country's exports become more competitive when its own currency depreciates, which could stimulate industries that are focused on exports. Thus, economic activity and domestic investment may be boosted, especially in industries with an eye toward global markets. Conversely, a depreciating currency may make imported capital goods and raw commodities more expensive. This may make production more expensive for domestic companies, which would discourage investment in some sectors of the economy. Furthermore, changes in energy prices can have an immediate effect on a company's cost of production, particularly if that company operates in an energy-intensive industry. Elevated energy costs can escalate operational costs, hence diminishing profit margins and, occasionally, discouraging investment. Similarly, large government spending on agriculture can increase competition for available funds, especially if it is supported by borrowing. This could lead to higher interest rates and crowds out private investment. If too many resources are devoted to agriculture, money may be taken away from more lucrative and dynamic industries such as manufacturing, services, or technology. The overall diversity and growth of the economy can be hampered by this misallocation.

Further, we plot the pointwise derivatives of exchange rate, energy prices and agriculture expenditure against agriculture value added, household consumption and domestic investment to capture the various marginal effects (see Fig. 1, Fig. 2, Fig. 3 respectively). The findings together with the robustness test using the dynamic ARDL simulation model confirm the results of the KRLS.

In terms of policy, we recommend creating government-funded insurance schemes to shield farmers from losses in revenue brought on by unfavorable fluctuations in exchange rates. For farmers, this can serve as a safety net. More specifically, to support households that are at risk from variations in currency rates, there is a need for bolstering the social safety nets that are presently in place in Nigeria. This includes targeted assistance programs, food subsidies, or cash transfer programs. In addition, the study recommends that businesses should employ financial instruments like options and future contracts to assist them hedge against exchange rate risks. This can offer some defence against unfavorable currency fluctuations.

On energy prices and agricultural spending effects, we recommend offering incentives to households and farmers to embrace renewable energy sources, like solar or wind power, for heating and agricultural usage, to mitigate the effects of energy prices and agricultural spending. This will lessen reliance on conventional energy sources and lessen the effects of changes in energy prices. In a similar vein, we advise investing money in value chains and agribusiness initiatives rather than just crop farming. This has the potential to raise the value contributed to agriculture, generate jobs and income and boost economic growth.

### 5.1 Limitation of the study

One key limitation of this study is its inability to fully capture and simulate the interactions between various policy types or the impact of unforeseen exogenous shocks, such as pandemics or geopolitical events, which could alter the correlations under examination. Future research will gain insights into resilience and adaptation tactics by developing models that can take external shocks into account and evaluate their effects on the interaction between exchange rates uncertainty, energy prices, sectoral spending, and their effects on agriculture value added, household consumption, and domestic investment.

## Data availability statement

The data that support the findings of this study is available from the authors of this paper upon reasonable request.

## CRediT authorship contribution statement

**Paul Terhemba Iorember:** Writing – review & editing, Writing – original draft, Investigation, Formal analysis, Data curation, Conceptualization. **Nora Yusma Mohamed Yusoff:** Writing – original draft. **Philip Terhemen Abachi:** Writing – original draft. **Ojonugwa Usman:** Writing – original draft. **Andrew Adewale Alola:** Writing – review & editing.

## Declaration of competing interest

The authors declare that they have no known competing financial interests or personal relationships that could have appeared to influence the work reported in this paper.
